This article has been retracted.

# Clinical Effect of Digital Subtraction Angiography Combined with Neurointerventional Thrombolysis for Acute Ischemic Cerebrovascular Disease and Its Influence on Vascular Endothelial Function and Oxidative Stress

**DOI:** 10.1155/2022/2777865

**Published:** 2022-08-09

**Authors:** Xuna Wang, Xuesong Zhang, Qingbo Guan, Kuiyang Wang

**Affiliations:** ^1^Department of Radiology, The Second Hospital of Dalian Medical University, Dalian City, 116023 Liaoning Province, China; ^2^Department of Invasive Technology, The Second Hospital of Dalian Medical University, Dalian City, 116023 Liaoning Province, China

## Abstract

**Objective:**

Ischemic cerebrovascular disease is a commonly seen vascular disorder in clinical practice. Given the difficulty of drug therapy to achieve ideal curative effects, interventional therapy has gradually become the preferred treatment for the disease. This research primarily discusses the short-term efficacy of digital subtraction angiography- (DSA-) guided neurointerventional thrombolysis for acute ischemic cerebrovascular disease (AICVD) and its influence on vascular endothelial function (VEF) and oxidative stress (OS).

**Methods:**

All the clinical data of 162 patients diagnosed with AICVD and treated between June 2019 and December 2021 were collected and analyzed retrospectively. They were assigned to two cohorts according to the difference in interventional methods: a conventional group (CG) given recombinant tissue plasminogen activator (rt-PA) therapy and an observation group (OG) intervened by DSA-guided neurointerventional thrombolysis. The two groups were compared with respect to short-term treatment efficacy, the National Institutes of Health Stroke Scale (NIHSS) score, cerebral hemodynamics, and VEF and OS indexes.

**Results:**

The short-term efficacy was better in OG (93.98%) than in CG (82.28%). After treatment, the NIHSS score decreased in both cohorts with obvious differences within the group at different time points, and the posttreatment NIHSS score was lower in OG as compared to CG. OG had higher *Q*_m_ and *V*_m_ while lower *W*_v_, *Z*_cv_, and *R*_v_ than CG. Higher endothelial-dependent flow-mediated dilatation (FMD) was observed in OG, as well as lower ankle-brachial index (ABI) and pulse wave velocity (PWV). And the posttreatment MDA was lower while SOD, GSH-Px, and TAC were higher in OG compared with those on CG. All the above differences were of statistical significance (*P* < 0.05).

**Conclusions:**

DSA-guided neurointerventional thrombolysis is highly effective in the treatment of AICVD, which can not only effectively improve patients' neurological function and cerebral hemodynamics but also mitigate VEF injury and help to alleviate patients' OS.

## 1. Introduction

As a common critical and severe condition worldwide, ischemic cerebrovascular disease (ICVD) refers to transient or persistent and local or diffuse brain tissue damage caused by ischemia and hypoxia of the corresponding brain tissue, resulting in a series of neurological dysfunction symptoms or signs [1, 2], with high disability rate and fatality rate [3, 4]. As the diet structure of people changes and the aging of the population accelerates, the prevalence of ICVD, most of which occurs on the basis of hemodynamic disturbance or cerebrovascular diseases, has increased rapidly, posing a serious threat to patients' life safety and quality [5, 6]. ICVD includes transient ischemic attacks (TIA) [7] and acute cerebral infarction (ACI) [8]. Regardless of the type, artery stenosis or occlusion caused by atherosclerosis is a very important reason [9].

Literature has revealed a close association between ICVD and atherosclerosis [10]. Ischemic cerebral vessels can cause temporary blood supply disturbance, resulting in neurological deficits, which have a serious impact on patients. Its onset is often accompanied by neurological dysfunction, and untimely treatment of the sudden attack of ICVD will seriously affect the life of patients. Thrombolysis is a commonly used clinical method to treat cerebral vascular occlusion and an important way to restore the patency of the occluded cerebral vessels [11]. The prominent feature of clinical treatment is intravenous (IV) thrombolysis (IVT). In thrombolytic drugs, plasminogen activators can dissolve fibrin in thrombi and promote the recanalization of blocked vessels, thus saving patients' lives in a timely manner [12–14]. However, IVT still has limitations. It only works within 4 hours after onset, with some certain contraindications for some patients [15]. Therefore, IVT, with limited therapeutic effectiveness, is not suitable for all cases. Interventional therapy, thanks to the progress of clinical medicine, has also been extensively applied, providing a new approach for cerebrovascular occlusion [16]. Interventional therapy is a minimally invasive method to determine the location of artery stenosis and treat cerebrovascular diseases through intubation based on computer. During interventional therapy, IVT can be used to dredge blood vessels and eliminate infarction [17], which has been confirmed by Liu et al. [18] and Lei et al. [19]. But the demerits of interventional therapy have also been gradually unveiled with its widespread application. The wrong choice of puncture site, for instance, can result in ineffective treatment while aggravating the patient's condition [20]. Due to the complexity of cerebrovascular structure, correct selection of the puncture site is critical. Hence, relevant auxiliary examination is the key to enhancing the treatment outcome of interventional therapy.

Digital subtraction angiography- (DSA-) guided neurointerventional thrombolysis is an operation assisted by imaging means, which can recanalize the lumen of the refractory occlusion or severe stenosis of cerebral blood supply artery through guidewires and catheters, and is widely used in clinic because of its advantages of small trauma, definite curative effect, and high safety [21, 22]. Besides, endothelial dysfunction (ED) in the cerebral circulation is shown to be linked to a range of vascular-related disorders, as well as a higher possibility of experiencing acute clinical events that may lead to cognitive decline [23–25]. Meanwhile, there is compelling evidence that oxidative stress (OS) is a major inducement of cerebral ED in multiple disorders [26]. Thus, this experiment primarily analyzes the therapeutic effect of DSA combined with neurointerventional thrombolysis on acute ischemic cerebrovascular disease (AICVD) patients and studies its effects on cerebral hemodynamics, vascular endothelial function (VEF), and OS, with the novelty and motivation lying in providing a scientific theoretical basis and laying a sound theoretical basis for further treatment.

## 2. Materials and Methods

### 2.1. General Data

We retrospectively analyzed the clinical data of 162 AICVD patients diagnosed and treated in the Second Hospital of Dalian Medical University between June 2019 and December 2021. Inclusive criteria: (1) all patients were confirmed by CT, MRI, and other imaging examinations and met the diagnostic criteria of AICVD [27]; (2) onset of illness ≤ 4.5 hours; (3) no previous interventional therapy; and (4) intact case data. Exclusion criteria: (1) presence of intracranial space-occupying lesions such as brain abscess and brain tumor, (2) severe organ dysfunction or diseases, (3) history of acute cerebral infarction or myocardial infarction within 3 months, (4) mental illness or cognitive impairment, (5) contraindications associated with other thrombolytic therapy and DSA antiplatelet drugs, and (6) incomplete case data. Patients were assigned to either the conventional group (CG; *n* = 79) or the observation group (OG; *n* = 83) based on the interventional methods. The comparison of baseline data (sex, age, etc.) showed no statistical difference between groups, suggesting clinical comparability (*P* > 0.05, Table 1). This study has obtained approval from the Medical Ethics Committee of the Second Hospital of Dalian Medical University. As this study was retrospective, the need for subjects' informed consent was waived.

### 2.2. Treatment Methods

All patients were monitored for vital signs after admission, and intracranial CT perfusion imaging and other auxiliary examinations were performed to determine the lesion site and the presence of cerebral hemorrhage. Among them, cases in OG were treated with DSA combined with neurointerventional thrombolysis. Recombinant tissue plasminogen activator (rt-PA) (alteplase for injection, specification 50 mg, Registration No. S20160055, Boehringer Ingelheim Pharma GmbH & Co. KG, Germany) was administered at 0.6 mg/kg intravenously, with the maximum dose controlled within 60 mg; 10% of the total dosage was first given via an IV bolus injection within 1 min, and the rest was pumped continuously within 1 h through the infusion pump. The Seldinger puncture technique was used to perform puncture, intubation, and arterial sheathing in the femoral artery of the patient, and a whole-brain DSA was performed to evaluate the vascular occlusion. The microguidewire was inserted, under whose guidance, the catheter was placed to the position near the diseased vessel. Then, a mixed solution of 200,000 U urease and 20 mL normal saline (0.9%) was quickly injected with a syringe, followed by pumping of 200,000 to 500,000 U urokinase and 50 mL normal saline (0.9%) with a microautolysis catheter at 1.0 mL/min. Patients in CG received conventional IV thrombolytic therapy with 0.9 mg/kg recombinant human tissue fibrinogen activator; 10% of the total dosage was first administered via an IV push within 1 min, and the rest was pumped continuously within 1 h through the infusion pump.

### 2.3. Endpoints

1. National Institutes of Health Stroke Scale (NIHSS) [28]: patients were assessed by the NIHSS score (score range: 0-45) before as well as 1 day, 7 days, and 3 months after treatment for neurological deficits, mainly from the dimensions of level of consciousness, response to commands, gaze, facial paralysis, motor function (leg), sensory, and dyskinesia. Higher scores were associated with more serious neurological deficits
2. Short-term efficacy: after 3 months of treatment, two physicians with deputy senior titles or above in the neurology department conducted efficacy assessment through the NIHSS score, with an inverse connection between the score and efficacy. Cure: NIHSS score lowered by >90%, with no disability. Marked response: NIHSS score lowered by 46%-90%, with basically independent living. Response: NIHSS score decreased by 18%-45%, with partial independent living ability. Nonresponse: NIHSS score decreased by less than 18%, with grade 3 or higher disability. Overall response rate (ORR) = (cure + marked response + response) cases/total cases × 100%
3. Cerebral hemodynamics: the cerebral blood flow of patients was measured using a CV-300 cerebrovascular hemodynamic analyzer (MEDENG Electronic Equipment Co., Shanghai, China). According to the empirical formula such as the basic equation of nonlinear elastic cavity model, several characteristic parameters reflecting cerebrovascular function were calculated by the computer system. The indexes measured before and after treatment included the mean blood flow (*Q*_m_), mean blood flow velocity (*V*_m_), wave velocity (*W*_v_), vascular characteristic impedance (*Z*_cv_), and peripheral resistance (*R*_v_)
4. VEF: the VEF of patients was measured with the use of an UNEXEF38g automated diagnostic ultrasound system (UNEX corporation, Sakae Naka-ku, Nagoya, Japan). The parameters detected before and after treatment included flow-mediated vasodilation (FMD), as well as bilateral ankle-brachial index (ABI) and brachial-ankle pulse wave velocity (ba-PWV) measured by a VBP-9 arteriosclerosis tester, and the average values of ABI and ba-PWV were calculated
5. OS: before and after treatment, fasting venous blood samples (4 mL) were obtained from each participant during morning hours, which were then treated with centrifugation (3000 r/min, 10 min) for serum collection. The enzyme-linked immunosorbent assay (ELISA) quantified serum total antioxidant capacity (TAC), and the xanthine oxidase method, thiobarbital colorimetry, and colorimetry determined malondialdehyde (MDA), superoxide dismutase (SOD), and glutathione peroxidase (GSH-Px), respectively

### 2.4. Statistical Processing

The sample size of this study was calculated using PASS 15.0 (NCSS, Kaysville, Utah). The data from a preliminary study indicated that for a study power of 80% (*α* = 0.05, *β* = 0.2), assuming an effective rate of 93% and 75% in OG and CG, respectively, the sample size required for each group was 62, with a total of 124 cases allowed for adequate data acquisition. Meanwhile, with the dropout rate of 20%, a total of 156 patients were needed (78 in each group).

All data were processed with SPSS 25.0 (SPSS, Inc., Chicago). The mean ± standard deviation was utilized to indicate the normal distributed quantitative data, and the intergroup and multigroup comparison methods were independent sample *t*-test and one-way analysis of variance plus Bonferroni post hoc analysis, respectively. Counting data were expressed by the case number (percentage), and the comparison adopted the chi-square test. Statistically significant differences were present when *P* < 0.05.

## 3. Results

### 3.1. NIHSS Scores of Two Groups

No statistical difference was found between OG and CG in pretreatment NIHSS scores. After treatment, decreased NIHSS scores were observed in both cohorts, with a statistical difference at each time point within the group (*P* < 0.05). And the NIHSS scores of OG were lower at 1 d, 7 d, and 3 months after treatment versus CG (*P* < 0.05), as exhibited in Table 2.

### 3.2. Clinical Efficacy of Two Groups

In CG, cure, marked response, response, and nonresponse were found in 13, 28, 24, and 14 cases, respectively, with an ORR of 82.28%. In OG, cure, marked response, response, and nonresponse were identified in 21, 38, 19, and 5 cases, respectively, with an ORR of 93.98%. The above data revealed a higher ORR in OG as compared to CG (*P* < 0.05), as can be found in Table 3.

### 3.3. Cerebral Hemodynamics in Two Groups

The intergroup comparison of pre- and posttreatment cerebral hemodynamics showed a statistically significant difference (*P* < 0.05). The posttreatment *Q*_m_, *V*_m_, *W*_v_, *Z*_cv_, and *R*_v_ in OG were 4.67 ± 1.10 mL/s, 12.77 ± 2.83 cm/s, 18.26 ± 4.26 m/s, and 82.12 ± 14.16 kPa·s/ms, and 53.60 ± 11.23 kPa·s/m, respectively; in CG, the corresponding indexes were 4.01 ± 0.65 mL/s, 10.78 ± 2.49 cm/s, 21.44 ± 4.81 m/s, 90.57 ± 17.47 kPa·s/m, and 59.56 ± 11.77 kPa·s/m, respectively. The results showed better recovery of cerebral hemodynamic indexes in OG compared with CG. See Table 4 for details.

### 3.4. VEF in Two Groups

Similarly, VEF differed significantly between groups before and after treatment (*P* < 0.05). The FMD, ABI, and PWV in OG were 5.88 ± 1.35%, 0.91 ± 0.10, and 1212.00 ± 50.82 cm/s/s after treatment, while those in CG were 5.16 ± 1.19%, 1.10 ± 0.11, and 1344.06 ± 68.82 cm/s, respectively, suggesting better recovery of VEF indexes in OG as compared to CG (*P* < 0.05). See Figure 1 for details.

### 3.5. OS Response in Two Groups

Serum SOD, MDA, GSH-Px, and TAC levels differed insignificantly between groups prior to treatment (*P* > 0.05). After treatment, serum SOD, GSH-Px, and TAC in the two groups all increased, while the content of MDA decreased, with statistically significant differences (*P* < 0.05); OG showed better improvement in each index than CG after treatment, as shown in Figure 2.

## 4. Discussion

In patients with ICVD, the atherosclerotic plaque shedding in the cerebral artery or neck artery leads to reduced blood supply to the brain, which causes local cerebral blood circulation disorders [29], eventually resulting in transient damage of varying degrees. During the clinical treatment of such patients, promoting blood supply restoration in the brain tissue and clearing blocked blood vessels is most frequently needed. Among them, thrombolytic therapy is a very common treatment, which is to dredge the blocked blood vessels, so that the blood and oxygen supply to the patient's brain tissues can be restored as soon as possible [30]. Among all kinds of thrombolytic therapy, neurointerventional therapy is minimally invasive, which uses guidewires, balloon dilatation, and other related materials to explore and treat the diseased blood vessels through intravascular catheters [31], while DSA can obtain clear and pure vascular images through subtraction, enhancement, and reimaging to achieve vascular visualization. The application of DSA in the process of implementing neurointerventional thrombolytic therapy can better relieve the stenosis and obstruction of diseased blood vessels, restore the blood perfusion of brain tissue, control the development of patients' condition, and effectively improve patient prognosis [32].

This study compared the short-term therapeutic efficacy, cerebral hemodynamics, VEF, and OS indexes of ICVD patients treated with conventional IVT and those with DSA-guided neurointerventional thrombolysis. The results showed a significantly higher ORR in patients receiving DSA combined with neurointerventional thrombolysis compared those with conventional IVT alone, similar to the research of Li et al. [33]. Besides, we found decreased NIHSS scores in both cohorts after treatment, especially in OG. Thrombolytic therapy can promote cerebral vascular recanalization and restore cerebral blood perfusion, which is conducive to relieving symptoms of neurological deficits and promoting patients' rehabilitation. As a targeted administration through guidewires and catheters under the support of DSA and other imaging means, neurointerventional thrombolysis can directly act on the diseased blood vessels and increase the contact area between thrombolytic drugs and thrombus, playing a positive role in promoting the recovery from neurological deficits. Further, we analyzed cerebral hemodynamics and found improvements in related indexes in both groups after treatment, suggesting improved blood supply of arterial vascular bed and significantly increased cerebral blood flow after thrombolytic therapy. Moreover, the improvement was more significant in OG, which indicates that neurointerventional thrombolysis on the basis of IVT is beneficial to improve cerebral hemodynamics, promote cerebral circulation recovery, and relieve the symptoms of ischemia, hypoxia, and neurological function damage. In the research of Yang et al. [34], insufficient blood supply to the brain would cause excessive lactic acid production and accumulation, resulting in acidosis, a process that is an important mechanism of neuronal damage. DSA-guided neurointerventional thrombolysis can effectively improve cerebral hemodynamics and blood circulation, which is conducive to early and adequate blood perfusion of reversible injured neurons and alleviation of ischemia and hypoxia, thus improving neurological function.

ED is the earliest event of inflammatory injury and vascular damage after ischemia reperfusion [35]. Following ischemia, endothelial cells and astrocytes produce numerous chemokines and cytokines that induce the expression of adhesion molecules on endothelial cells, causing leukocyte adhesion and degrading endothelial tight junction proteins and extracellular matrix [36]. Therefore, inhibiting this inflammatory reaction can reduce ischemic infarct size and alleviate neurological deficits. In this study, FMD increased statistically while ABI and PWV decreased obviously after treatment in the two groups, with more significant changes in OG. FMD is an effective index to reflect the structural and functional integrity of vascular endothelial cells [37]; ABI and PWI can be used to predict the risk of atherosclerosis. The higher the ABI and PWI, the worse the vascular elasticity, and the greater the probability of developing atherosclerosis and cerebrovascular events [38]. In addition, OS is the main factor causing nerve injury after cerebral infarction [39], which is mainly manifested by increased lipid peroxidation products like MDA and reduced antioxidant enzymes like SOD, GSH-Px, and TAC, leading to increased blood vessel and cell permeability, inducing OS reaction and causing serious impact on nerve cell function. OS plays an important part in acute ischemic stroke pathogenesis [40]. In acute cerebral infarction, oxygen uptake in brain tissue is insufficient to maintain cellular oxidative metabolism, causing metabolic changes and cell death. The brain, for many reasons, is particularly vulnerable to free radical injury. The brain is rich in polyunsaturated fatty acids, which are particularly susceptible to free radical-induced peroxidation that alters the content of antioxidant enzymes [41]. This research identified lower MDA and higher SOD, GSH-Px, and TAC in OG compared with CG. It suggests that DSA-guided neurointerventional thrombolysis has obvious advantages in improving VEF, which is conducive to restoring vascular endothelial cell structure and function, promoting vasodilation, and increasing cerebral blood supply and flow. At the same time, it downregulates lipid peroxide expression, promotes oxygen free radical scavenging, and relieves oxidative damage to brain tissue, contributing to reduced OS and accelerated neurological recovery.

## 5. Conclusion

To sum up, for the treatment of AICVD, DSA combined with neurointerventional thrombolysis can effectively improve cerebral hemodynamics, reduce VEF damage, alleviate the body's OS response, and promote the recovery of nerve function, which has high clinical popularization value. However, further in-depth research is needed to explore the interaction between DSA and neurointerventional thrombolysis. Besides, the key action sites of the treatment are still being explored. There is still a long way to go for the wide clinical application of adverse reactions after treatment, and the benefits and risks of treatment should be effectively weighed to ensure the clinical treatment effect.

## Figures and Tables

**Figure 1:** Comparison of vascular endothelial function. (a) Comparison of FMD; (b) comparison of ABI; (c) comparison of PWV; ^∗^*P* < 0.05*vs.* the conventional group before treatment; ^#^*P* < 0.05*vs*. the observational group before treatment; ^∗∗^*P* < 0.01 and ^∗∗∗^*P* < 0.001.

**Figure 2:** Comparison of oxidative stress indexes. (a) Comparison of SOD; (b) comparison of MDA; (c) comparison of GSH-Px; (d) comparison of TAC; ^∗^*P* < 0.05*vs.* the conventional group before treatment; ^#^*P* < 0.05*vs*. the observational group before treatment; ^∗∗∗^*P* < 0.001.

**Table 1:** Comparison of general data.

	Conventional group (*n* = 79)	Observation group (*n* = 83)	*χ* ^2^/*t*	*P*
Gender (*n*)			1.2481	0.2639
Male	45 (57.0)	40 (48.2)		
Female	34 (43.0)	43 (51.8)		
Age (years old)	50.52 ± 10.14	50.76 ± 10.23	0.1499	0.8810
Body mass (kg)	61.60 ± 7.32	62.87 ± 8.10	1.0453	0.2975
Primary disease (*n*)				
Diabetes mellitus	19 (24.1)	24 (28.9)	0.4913	0.4833
Hypertension	37 (46.8)	40 (48.2)	0.0299	0.8627
Hyperlipidemia	35 (44.3)	38 (45.8)	0.0358	0.8500
History of smoking (*n*)	39 (49.4)	39 (47.0)	0.0918	0.7619
History of drinking (*n*)	23 (29.1)	28 (33.7)	0.4007	0.5267

**Table 2:** Comparison of NIHSS scores.

	Before treatment	1 d after treatment	7 d after treatment	3 months after treatment	*F*	*P*
Conventional group (*n* = 79)	21.05 ± 4.31	13.59 ± 2.62	8.00 ± 1.64	6.29 ± 1.27	470.4000	<0.0001
Observation group (*n* = 83)	21.39 ± 3.94	10.66 ± 2.68	6.23 ± 1.26	4.42 ± 0.91	765.2000	<0.0001
*t*	0.5244	7.0318	7.2515	10.8124	—	—
*P*	0.60007	<0.0001	<0.0001	<0.0001	—	—

**Table 3:** Comparison of clinical efficacy.

	Cure	Marked response	Response	Nonresponse	Overall response rate
Conventional group (*n* = 79)	13 (16.46)	28 (35.44)	24 (30.38)	14 (17.72)	65 (82.28)
Observation group (*n* = 83)	21 (25.31)	38 (45.78)	19 (22.89)	5 (6.02)	78 (93.98)
*χ* ^2^					4.5871
*P*					0.0322

**Table 4:** Comparison of cerebral hemodynamic indexes.

Time point	Groups	*Q*_m_ (mL/s)	*V*_m_ (cm/s)	*W*_v_ (m/s)	*Z*_cv_ (kPa·s/m)	*R*_v_ (kPa·s/m)
Before treatment	Conventional group (*n* = 79)	3.36 ± 0.77	8.13 ± 2.26	25.10 ± 4.72	146.82 ± 20.38	84.17 ± 13.85
	Observation group (*n* = 83)	3.20 ± 0.80	8.26 ± 2.24	25.96 ± 4.46	146.34 ± 24.32	83.20 ± 15.97
*t*		1.2959	0.3676	1.1924	0.1358	0.4121
*P*		0.1969	0.7136	0.2349	0.8921	0.6808
After treatment	Conventional group (*n* = 79)	4.01 ± 0.65^∗^	10.78 ± 2.49^∗^	21.44 ± 4.81^∗^	90.57 ± 17.47^∗^	59.56 ± 11.77^∗^
	Observation group (*n* = 83)	4.67 ± 1.10^#^	12.77 ± 2.83^#^	18.26 ± 4.26^#^	82.12 ± 14.16^#^	53.60 ± 11.23^#^
*t*		4.6198	4.7423	4.4597	3.3896	3.2982
*P*		<0.0001	<0.0001	<0.0001	0.0008	0.0011

Notes: ^∗^*P* < 0.05*vs*. the conventional group before treatment; ^#^*P* < 0.05*vs*. the observational group before treatment.

## Data Availability

The labeled dataset used to support the findings of this study is available from the corresponding author upon request.
